# Analysis of Related Factors Affecting Facial Nerve Function after Acoustic Neuroma Surgery

**DOI:** 10.1155/2022/5194566

**Published:** 2022-08-09

**Authors:** Chunhan Liu, Yage Shen, Dongyi Han, Di Zhang

**Affiliations:** ^1^Vertigo Clinic, The Third People's Hospital of Shenzhen, Shenzhen 518000, China; ^2^Department of Otolaryngology, The Third People's Hospital of Shenzhen, Shenzhen 518000, China; ^3^Baoding No. 1 Hospital of TCM, Baoding 071000, China; ^4^College of Otolaryngology Head and Neck Surgery, Chinese People's Liberation Army General Hospital, Chinese People's Liberation Army Medical School, National Clinical Research Center for Otolaryngologic Diseases, State Key Lab of Hearing Science, Ministry of Education, Beijing 100853, China

## Abstract

**Objective:**

To investigate the factors affecting facial nerve function after acoustic neuroma surgery and to provide theoretical reference for clinicians to preserve facial nerve function better after surgery.

**Methods:**

A retrospective cohort study was conducted to analyze the correlation between postoperative facial nerve function and surgical approach, age, sex, tumor size and adhesion degree of facial nerve in 152 patients with acoustic neuroma.

**Results:**

In the choice of surgical approach, there was no significant difference in the anatomy of the complete facial nerve in labyrinth path, retrosigmoid sinus path, and middle cranial fossa path. There was no statistically significant difference between the middle cranial fossa path and the retrosigmoid sinus path in facial nerve function preservation 7 days after surgery. The difference between middle cranial fossa path and labyrinthine path was statistically significant (*P* < 0.01). There were statistically significant differences between labyrinth path and retrosigmoid sinus path (*P* < 0.05). Logistic multivariate regression analysis showed that the operative approach and the degree of adhesion between tumor and facial nerve were the risk factors affecting functional preservation of facial nerve 7 days after surgery. Age and the degree of adhesion between tumor and facial nerve were the risk factors for functional preservation of facial nerve 1 year after operation.

**Conclusion:**

The facial nerve function injury in patients with acoustic neuroma may be related to the choice of surgical approach, the adhesion degree of tumor and facial nerve, and their age. Clinicians need to comprehensively evaluate the risk factors before surgery, so as to achieve individualized treatment to protect the integrity of postoperative facial nerve function of patients.

## 1. Introduction

Acoustic neuroma, also known as vestibular schwannoma, originates from the eighth cranial nerve sheath and is the third benign tumor with the highest incidence among intracranial tumors [1], accounting for about 80%–90% of pontine angle tumors. Patients with hearing loss, tinnitus, vertigo, earache, facial numbness, skin paresthesia, and drinking water cough as the main symptoms. Growing tumors can compress the lateral pons and the frontal cerebellum and even endanger the patient's life in severe cases. At present, the main treatment strategies for this disease are follow-up observation, microsurgical resection, stereotactic radiotherapy, etc. Compared with the other two groups of treatment strategies, surgical resection can effectively reduce tumor volume and solve complications [2, 3] and greatly improve the postoperative quality of life of patients. Therefore, surgery is now widely accepted by both doctors and patients as the preferred method.

In recent years, with the development of microsurgical technology and the wide application of intraoperative facial nerve monitoring technology, the mortality rate of acoustic neuroma surgery in the world has decreased sharply, and the therapeutic target has entered a new stage of preserving facial nerve function. Although intraoperative facial nerve protection and tumor resection extent are improved, different rates of neuroanatomical preservation and functional preservation have occurred [4]. Therefore, the purpose of this study is to investigate the possible factors related to the influence of facial nerve function after acoustic neuroma surgery in order to provide some theoretical reference for the clinical diagnosis and treatment.

## 2. Materials and Methods

### 2.1. Research Objects

Patients diagnosed with acoustic neuroma and treated with surgery in the General Hospital of the Chinese People's Liberation Army from January 2004 to August 2015 were collected.

#### 2.1.1. Inclusion Criteria

1. After admission, pure tone audiometry, speech recognition rate, acoustic impedance test, auditory brainstem response, otoacoustic emission, and vestibular function examination were performed;
2. the patient was diagnosed as acoustic neuroma by preoperative temporal bone CT and cranial MRI and confirmed as acoustic neuroma by postoperative pathological results;
3. all patients' surgeries were completed by the same team;
4. patients and their families signed informed consent before surgery.

#### 2.1.2. Exclusion Criteria

1. Previous history of lateral skull base surgery;
2. the patient had received stereotactic radiotherapy;
3. facial nerve disorder before operation namely.

### 2.2. Methods

In this study, patients' age, gender, surgical approach, tumor size, and the degree of adhesion between tumor and facial nerve were collected retrospectively. Facial nerve function was recorded 7 days after surgery and 1 year after surgery by way of follow-up.

#### 2.2.1. Intraoperative Facial Nerve Monitoring Methods

Facial nerve monitoring uses the nerve recognition monitor developed by the American Medtronic Company. After the patients were satisfied with general anesthesia, three pairs of needle-like electrodes were placed on the forehead, upper lip, and superior sternal fossa on the operative side, and fixed with adhesive film. During the operation, the stimulation probe of the facial nerve monitor was used to touch and detect the location of the facial nerve according to the size of the monitoring sound induced by the facial muscle convulsion when the facial nerve was stimulated by the electric current.

#### 2.2.2. Facial Nerve Function Retention Assessment Method

Three senior audiologists used the house-Brackmann (HB) facial nerve function grading method to subjectively evaluate the facial nerve function of the patients 7 days and 1 year after surgery. HB I–II was defined as good facial nerve function, III–IV as moderate facial nerve function, and V–VI as poor facial nerve function. The grade of facial nerve function was assessed and recorded statistically according to 2 : 1.

#### 2.2.3. Statistical Methods

SPSS (V.17.0) software was used for statistical analysis. The counting data are represented by *n* and %. A mean ± SD was used for data consistent with normal distribution in measurement data, and a Wilcoxon rank sum test was used for comparison of continuity variables between the two groups. A logistic regression model was used to analyze the correlation between facial nerve function preservation and surgical approach, tumor size, age, gender, and the degree of adhesion between tumor and facial nerve. *P* < 0.05 means the difference is statistically significant.

## 3. Results

### 3.1. Basic Data of Patients

A total of 152 cases of acoustic neuroma were resectomized under facial nerve monitoring, including 69 males and 83 females, ranging in age from 13 to 71 years, with an average age of 42.08 ± 12.48 years. The tumors were classified according to the size and stage: 13 cases of stage I auditory type, 17 cases of stage II small, 68 cases of stage III medium, 46 cases of stage IV large, and 8 cases of stage V giant. The degree of adhesion between the tumor and the facial nerve was evaluated according to what the surgeons saw during the operation. There were 43 cases without adhesion, 44 cases with mild adhesion, 35 cases with moderate adhesion, and 30 cases with severe adhesion. Among the surgical approaches, 96 were via the retrosigmoid sinus, 49 were via the labyrinth, and 7 were via the middle cranial fossa (see Table 1).

### 3.2. Facial Nerve Anatomy and Functional Retention Data of Patients

The basic condition that acoustic neuroma operation retains facial nerve function is to retain the integrality of facial nerve anatomy. 145 patients with intact facial nerve anatomy were studied. 2 cases were interrupted via the labyrinth path and 5 cases were interrupted via the retrosigmoid sinus. The interrupted patients underwent sublingual anastomosis of the facial nerve or facial nerve diversion anastomosis at the same time (see Table 2).

(Patients with intraoperative severance of the facial nerve were subjected to nerve anastomosis, and the phenomenon was considered as intraoperative injury to the facial nerve, and their facial nerve function at 7 days and 1 year after surgery was incorporated into Table 3 and 4).

According to the house-Brackmann (HB) facial nerve function grading method, the facial nerve function reached HB Grade I–II in 98 patients, grade III–IV in 51 patients, and grade V–VI in 3 patients 7 days after the operation. Facial nerve function reached HB Grade I–II in 131 cases, III–IV in 20 cases, and V–VI in 1 case one year after operation (see Tables 5 and 6).

### 3.3. Surgical Approach Analysis Results

The facial nerve anatomical integrity of the labyrinth path, sigmoid sinus path, and middle cranial fossa path was compared by pairwise group, and the differences were not statistically significant (see Table 7).

Facial nerve function of each surgical approach 7 days after surgery and 1 year after surgery are shown as follows (see Tables 3 and 4).

Through counting the facial nerve functions to 7 days after the operation for the three surgical approaches, we found no significant difference between the middle cranial fossa path compared with the rectosigmoid sinus path, but there was a significant difference between the two surgical approaches mentioned above compared with the labyrinth path. There was no significant difference in facial nerve function among the three groups in pairs one year after operation (see Tables 8 and 9).

### 3.4. Results of Multifactor Analysis

Gender, age, surgical approach, tumor size, and degree of adhesion between tumor and facial nerve were analyzed by logistic multifactor regression at 7 days and 1 year after acoustic neuroma. The results showed that the operative approach and the degree of adhesion between tumor and facial nerve were the risk factors affecting facial nerve function 7 days after the operation. Age and the degree of adhesion between the tumor and the facial nerve are related risk factors that affect facial nerve function one year after operation (see Tables 10 and 11).

## 4. Discussion

At present, the treatment expectation for acoustic neuroma is to completely remove the tumor and retain the intact facial nerve function [5], so as to avoid facial nerve function injury to different degrees of facial regional paralysis as much as possible, which will bring many adverse effects to the postoperative life and work of patients. In this study, the facial nerve anatomical retention rate of acoustic neuroma surgery was 95.4% (145/152); the proportion of facial nerve function reaching grade I–II was 64.5% (98/152) 7 days after surgery; and 86.2% (131/152) 1 year after surgery. Facial nerve anatomical retention rate and functional retention rate are different, and it is still difficult to maintain the functional integrity of the facial nerve after surgery [6]. Therefore, it is essential to fully understand the relevant factors affecting facial nerve functional retention.

Acoustic neuroma often occurs in the trigone of the pontine cerebellum, which is accompanied by many important blood vessels and nerves and is closely linked with the pons, cerebellum, posterior cranial nerves and other structures. The main surgical approaches for auditory neuroma were the posterior sigmoid sinus approach, the middle cranial fossa approach, and the vagus approach. This study found that the preservation of facial nerve function at 7 days postoperatively via the vagus approach was better than the other two approaches, presumably with a lesser degree of damage to the facial nerve in the former group. According to literature reports, current neurosurgeons are good at using the retrosigmoid sinus path for surgery because of its wide application scope, high tumor resection rate, and early recognition of the facial nerve path [7]. However, with the continuous development of ear microsurgery and facial nerve monitoring systems, labyrinthine pathway gradually highlights its main advantages, namely, less surgical risk. The direct resection of the tumor can be carried out with early positioning and exposure of the facial nerve, which greatly reduces the facial nerve's touching, pulling, and other harassment. In recent years, the therapeutic scope of modified surgery is no longer limited to small acoustic neuromas [8, 9] so more clinicians have chosen it. Because the facial nerve anatomical integrity of the three surgical approaches was roughly the same during the operation, and facial nerve edema and other problems that occurred during the operation could be resolved and repaired with the passage of time, there was no significant difference in the effect of different surgical approaches on the facial nerve function one year after the operation.

In this study, age was one of the relevant factors affecting facial nerve function 1 year after surgery but not 7 days after surgery. The reason for this result may be related to the decrease of nerve growth factor level year by year and facial nerve edema after surgery, because nerve growth factor can effectively regulate the growth and repair of neurons in the nervous system [10]. According to literature reports, nerve growth factor has a protective effect on ototoxic neural deafness, which can promote the survival and differentiation of mouse neural stem cells and upregulate the excitability of nerve cells [11]. In addition, its concentration has a certain time characteristic in the mouse intracranial [12]. Therefore, we speculated that with the increase of patients' age, the concentration of growth factors of the nutritional facial nerve decreases, thus affecting the recovery rate of the body. However, at present, there are differences on whether age affects postoperative facial nerve function, and some scholars [13, 14] put forward contradictory research conclusions. Postoperative facial nerve edema may be related to intraoperative harassment. The facial nerve dysfunction caused by such acute injury was not affected by the age of the patient. As long as the facial nerve anatomical structure was intact during the operation, the symptoms of postoperative facial paralysis could be gradually improved [15].

This study found that whether 7 days or 1 year after surgery, functional retention of the facial nerve was correlated with the degree of adhesion between the tumor and the facial nerve. Studies have confirmed that the degree of adhesion between tumor and facial nerve is an important factor affecting the integrity of facial nerve preservation [16, 17]. In clinical observation, the acoustic neuroma of nerve fibroma disease II often infiltrates facial nerve, but pure acoustic neuroma also exists adherent to the circumstance at facial nerve. Intraoperative separation of mild adhesions can preserve the integrity of the nerve and arachnoid. Moderate adhesions may damage the nerve, and severe adhesions may lead to separation of nerve fibers [16]. Although Hou [18] believed that small acoustic neuromas rarely infiltrate the facial nerve, this conclusion could not be applied to all patients. At present, it is believed that the adhesion degree of small tumor and facial nerve can also directly affect the surgical effect [19]. The higher the degree of adhesion between the tumor and the facial nerve, the higher the probability of damage to the facial nerve caused by intraoperative separation. Based on the results of the correlation between tumor size and facial nerve function retention in this study, it is presumed that the former has a more direct effect.

In conclusion, surgical approach and the degree of adhesion between tumor and facial nerve are related risk factors affecting functional preservation of the facial nerve 7 days after surgery. Age and the degree of adhesion between tumor and facial nerve were the risk factors for functional preservation of the facial nerve 1 year after operation. Incorrect surgical approach, older age, and higher degree of adhesion between tumor and facial nerve increase the risk of postoperative facial nerve functional injury, and the patient's recovery ability is reduced. The above results suggest that clinicians need to comprehensively evaluate the patient's risk factors before acoustic neuroma surgery, select appropriate surgical methods, and achieve individualized treatment to protect the postoperative facial nerve function integrity and improve the postoperative quality of life of patients.

## Figures and Tables

**Table 1:** Basic data of patients.

Project	Category	Cases (*n*)	Percentage (%)
Gender	Male	69	45.4
	Female	83	54.6
Tumor size	Stage I auditory type	13	8.6
	Stage II small	17	11.2
	Stage III medium	68	44.7
	Stage IV large	46	30.3
	Stage V giant	8	5.3
The degree of tumor and facial nerve adhesion	No adhesion	43	28.3
	Mild adhesion	44	28.9
	Moderate adhesion	35	23.1
	Severe adhesion	30	19.7
Surgical approach	Retrosigmoid sinus path	96	63.2
	Labyrinth path	49	32.2
	Middle cranial fossa path	7	4.6

**Table 2:** The anatomy of three kinds of surgical approaches.

Facial nerve anatomy	Retrosigmoid sinus path	Labyrinth path	Middle cranial fossa path
Integrated	47	7	91
Interrupted	2	0	5

**Table 3:** Facial nerve function 7 days after operation of three surgical approaches.

HB grade	Middle cranial fossa path	Labyrinth path	Retrosigmoid sinus path
I–II	1	41	56
III–IV	6	6	36
V–VI	0	2	4

**Table 4:** Facial nerve function 1 year after operation of three surgical approaches.

HB Grade	Middle cranial fossa path	Labyrinth path	Retrosigmoid sinus path
I–II	5	45	81
III–IV	2	4	14
V–VI	0	0	1

**Table 5:** Facial nerve function 7 days after operation.

HB grade	Cases (*n*)	Percentage (%)
I–II	98	64.5
III–IV	51	33.6
V–VI	3	1.9

**Table 6:** Facial nerve function 1 year after operation.

HB grade	Cases (*n*)	Percentage (%)
I–II	131	86.2
III–IV	20	13.1
V–VI	1	0.7

**Table 7:** Comparison of facial nerve anatomy of three surgical approaches.

Grouping	Rank sum difference	0.05 boundary value	0.01 boundary value	*P* value
Middle cranial fossa path vs. Labyrinth path	3.10	15.81	19.60	>0.05
Middle cranial fossa path vs. Retrosigmoid sinus path	3.96	15.32	18.99	>0.05
Labyrinth path vs. Retrosigmoid sinus path	0.86	6.87	8.52	>0.05

**Table 8:** Comparison of facial nerve function 7 days after operation with three surgical approaches.

Grouping	Rank sum difference	0.05 boundary value	0.01 boundary value	*P* value
Middle cranial fossa path vs. Labyrinth path	49.55	36.44	45.18	<0.01
Middle cranial fossa path vs. Retrosigmoid sinus path	31.03	35.31	43.78	>0.05
Labyrinth path vs. Retrosigmoid sinus path	18.52	15.83	19.63	<0.05

**Table 9:** Comparison of facial nerve function 1 year after operation with three surgical approaches.

Grouping	Rank sum difference	0.05 boundary value	0.01 boundary value	*P* value
Middle cranial fossa path vs. Labyrinth path	15.41	26.04	32.28	>0.05
Middle cranial fossa path vs. Retrosigmoid sinus path	9.67	25.23	31.28	>0.05
Labyrinth path vs. Retrosigmoid sinus path	5.74	11.31	14.03	>0.05

**Table 10:** Influencing factors of facial nerve function 7 days after operation.

Parameter	Estimated value	Standard error	*U*-value	*P* value	OR	95% CI
Constant term	−6.473	1.438	4.500	≤0.001		
Age	0.022	0.016	1.373	0.170	1.02	0.991∼1.005
Gender	0.730	0.399	1.829	0.067	2.07	0.949∼4.533
Tumor size	0.239	0.204	1.175	0.240	1.27	0.852∼1.894
The degree of tumor and facial nerve adhesion	0.559	0.201	2.783	0.005	1.75	1.180∼2.594
Surgical approach	1.332	0.391	3.403	0.001	3.79	1.759∼8.158

**Table 11:** Influencing factors of facial nerve function 1 year after operation.

Parameter	Estimated value	Standard error	*U*-value	*P* value	OR	95% CI
Constant term	−8.533	2.171	3.930	≤0.001		
Age	0.067	0.026	2.563	0.014	1.07	1.016∼1.126
Gender	-3.000	0.545	0.549	0.583	0.74	0.254∼2.158
Tumor size	0.214	0.289	0.741	0.458	1.24	0.703∼2.182
The degree of tumor and facial nerve adhesion	0.972	0.331	2.941	0.003	2.64	1.383∼5.052
Surgical approach	1.027	0.540	1.904	0.057	2.79	0.970∼8.043

## Data Availability

The data and materials during the current study are available from the corresponding author on reasonable request.
